# Comprehensive Analysis Identifies COL1A1, COL3A1, and POSTN as Key Genes Associated with Brain Metastasis in Patients with Breast Cancer

**DOI:** 10.1155/2022/7812218

**Published:** 2022-08-12

**Authors:** Weidan Wu, Linlin Zheng

**Affiliations:** Oncology Department, The Affiliated Hospital of Putian University, Putian, China

## Abstract

**Objective:**

Brain metastasis (BM) is associated with a high mortality in patients with breast cancer (BC). Nevertheless, the molecular mechanisms of BM in BM remain uncertain. The study aims to identify the key genes in BC in relation to BM and to assess their prognostic value.

**Methods:**

Two microarray datasets GSE125989 and GSE100534 were downloaded from the Gene Expression Omnibus (GEO) database to identify differentially expressed genes (DEGs) between primary BC and BM samples. The function enrichment analysis and protein-protein interaction (PPI) network were performed. We mapped hub genes into the Kaplan–Meier database for their correlations with BC survival.

**Results:**

Venn diagram analysis showed an overlapped upregulated DEG and 18 overlapped downregulated ones between primary BC and BM samples. We constructed the PPI network, and top 5 hub genes were sorted out according to the node degree, including type I collagen *α*_1_ chain (COL1A1), lumican (LUM), type III collagen *α*_1_ chain (COL3A1), type V collagen *α*_2_ chain (COL5A2), and periosteal protein (POSTN). The Kaplan–Meier database analysis found that COL1A1, COL3A1, and POSTN were significantly correlated with overall survival of BC patients.

**Conclusion:**

The study suggests that COL1A1, COL3A1, and POSTN may be key genes associated with BM in patients with BC.

## 1. Introduction

Breast cancer (BC) is one of the most common cancers in women, with a high incidence rate in female malignant tumors, ranking the second among the causes of cancer-related deaths in women [1]. Approximately, 4,820,000 and 2,370,000 populations were newly diagnosed with BC in China and USA in 2022, respectively, causing 3,210,000 and 640,000 deaths [2]. A large number of people have been diagnosed with advanced BC at the time of the first examination as a result of weak consciousness of cancer prevention and complex clinical characteristics [3]. Patients with advanced BC are usually accompanied by cancer metastasis. The central nervous system is one of the most common metastatic sites of BC. Brain metastasis (BM) of BC accounts for 15–30% of patients with breast cancer metastasis [4]. BC is responsible for primary causes of BM after lung cancer, accounting for 15% of BM [5]. Other primary cancers, such as lung, melanoma, and colorectal, most frequently metastasize to the brain, with estimated 45%, 10%, and 5% of BM, respectively [6]. Few therapeutic options are available for BC patients with BM, leading to poor prognosis and an estimated 1-year survival rate of 20% [7]. Recent studies have revealed that surgical resection of BM is considered as a standard treatment in prolonging survival, overall surgical mortality ranges from 0.7 to 1.9%, and neurological related diseases account for 3.9–6% of deaths. However, this resection is only suitable for appropriately selected patients with easily accessible metastatic sites, normal functions, nonextracranial diseases, or controllable extracranial diseases [8]. Of note, surgical resection is not an ideal scheme due to complications, such as postoperative seizures [9], urinary infections, and venous thrombosis [10]. In view of the poor prognosis and limited treatments for BC patients with BM, seeking for its mechanism is extremely important for early diagnosis and clinical treatments.

Previous studies have shown that proteins expressed in some metastatic primary BC cells contributed to the occurrence and development of BM before BC cells reached the brain. For instance, overexpression of antiplasminogen activator serpins, including neuroserpin and serpin B2, in metastatic BC cells promoted BM [11]. *α*B-crystallin expression in primary BC was related to poor overall survival and *α*B-crystallin silencing suppressed BM [12]. The mechanism of BC cell invasion and metastasis to the central nervous system remains unclear. In this study, we used Gene Expression Omnibus (GEO) datasets to screen overlapping differentially expressed genes (DEGs) between BC and BM samples and carried out the Kaplan–Meier plotter online database to identify hub genes related to prognosis. This may help to find out novel diagnostic biomarkers of BC with BM and provide evidence in clinical treatments.

## 2. Methods

### 2.1. Retrieval of the Microarray Dataset

Gene expression profiles between primary BC samples and BM samples were downloaded from the GEO database that is a subtool of the National Center for Biotechnology Information (NCBI). Firstly, the term “breast cancer brain metastasis” as a keyword was entered into the search box “Keyword or GEO Accession,” followed by selecting “Homo sapiens” as the specimen. Two datasets, GSE125989 and GSE100534, were chosen for differential expression analysis. The GSE125989 dataset contained tissue-derived RNA samples from 16 pairs of matching primary BC and BM, which was generated in the GPL571 platform. The GSE100534 dataset included tissue-derived RNA samples from 16 cases of primary BC and 3 cases of BM, which was generated in the GPL6244 platform. The raw data of two datasets were handled, normalized, and log2-transformed. The Limma package loaded in R/Bioconductor software, with |log2 (fold change [FC])| > 1.5 and corrected *P* value <0.05 as threshold values, was used to sort out DEGs.

### 2.2. Venn Analysis

Venn constructed diagrams of up to five simply connected regions that overlapped each other once in each possible way of overlapping. Venn intersect function was carried out for the purpose of obtaining overlapping DEGs between GSE125989 and GSE100534 datasets. Overlapping DEGs were regarded as final DEGs between primary BC and BM.

### 2.3. GO and KEGG Analyses of DEGs

The GO database offers comprehensive functional annotation tools to describe gene and gene product attributes in organisms (https://www.geneontology.org), and proteins can have multiple functional annotations in GO as one protein can perform multiple biological roles involving biological process (BP), cellular component (CC), and molecular function (MF). KEGG is a public online system database with a plethora of information on genomes, biological pathways, drugs, and chemical substances, in which gene networks and molecular networks were systematically analyzed. The Database for Annotation, Visualization, and Comprehensive Discovery (DAVID) was used to identify significantly GO terms and KEGG pathways enriched by genes, with a *P* value <0.05 by Fisher's exact test as a threshold value.

### 2.4. Protein-Protein Interaction (PPI) Network Construction and Hub Gene Screening

A PPI network was constructed to identify the functional interactions between predictive proteins and known proteins via the Search Tool for the Retrieval of Interacting Genes (STRING online tool). Hub genes were sorted out according to the node degree and the network of functional interaction between target genes and other genes. In theory, the more the connections, the more important the gene, indicating its wider associations with other genes. The PPI network was visualized using Cytoscape V3.7.3 software.

### 2.5. Prognostic Values of Hub Genes

The Kaplan–Meier plotter online database (https://kmplot.com/analysis/) was utilized to estimate the prognostic effects of the expression of 30,000 genes (mRNA, miRNA, protein) on patient survival in 25,000 samples from 21 tumor types covering breast, ovarian, lung, and gastric cancer on the basis of gene arrays, RNA-sequence, or next generation sequencing (for mutation data) and sourced from the databases including GEO, European Genome-phenome Archive (EGA), and The Cancer Genome Atlas (TCGA). In this study, the DEGs between primary BC and BM were mapped into the Kaplan–Meier database for their correlations with BC survival, with a log-rank test and a 95% hazard ratio (HR) calculated.

## 3. Results

### 3.1. Identification of DEGs in BC Associated with BM

We differentially analyzed the gene expression profiles of BC patients in the two microarray datasets, GSE125989 and GSE100534. After analyzing the GSE125989 dataset, we identified 58 downregulated DEGs and 4 upregulated DEGs between primary BC and BM samples, fulfilling |log_2_FC| > 1.5, and adjusted *P* < 0.05 (Figure 1(a)). After analyzing the GSE100534 dataset, we screened out 486 downregulated DEGs and 575 upregulated DEGs between primary BC and BM samples, fulfilling |log_2_FC| >1.5, and adjusted *P* < 0.05 (Figure 1(b)). Further Venn diagram analysis showed 19 overlapped DEGs containing an overlapped upregulated DEG and 18 overlapped downregulated ones (Figure 2(a)) listed below: COL1A1 (down), DPT (down), GREM1 (down), CILP (down), POSTN (down), IGF1 (down), COL3A1 (down), THBS2 (down), COL14A1 (down), LUM (down), ACTA2 (down), COL6A3 (down), LRRC15 (down), CCL19 (down), MMP11 (down), COL5A2 (down), AOX1 (down), KRT14 (down), and GAP43 (up).

### 3.2. Functional Enrichment Analysis of DEGs

Next, we conducted GO annotation and KEGG pathway analyses to assess the main functional terms and pathways of 19 overlapped DEGs between primary BC and BM samples. It was revealed by GO analysis that the DEGs between primary BC and BM samples were enriched in 66 GO terms (*P* < 0.05), covering 52 terms belonging to BP, 10 terms to CC, and 4 terms to MF (Figure 2(b), top 10 terms of BP presented). The KEGG pathway analysis identified 6 pathways significantly enriched by DEGs between primary BC and BM samples (*P* < 0.05) including protein digestion and absorption, focal adhesion, ECM-receptor interaction, the relaxin signaling pathway, the PI3K-Akt signaling pathway, and proteoglycans in cancer (Figure 2(c)).

### 3.3. Identification of Hub Genes

We mapped 19 overlapped DEGs between primary BC and BM samples into the STRING online tool to construct a PPI network (Figure 3), and top 5 hub genes were sorted out according to the node degree, including type I collagen *α*_1_ chain (COL1A1), lumican (LUM), type III collagen *α*_1_ chain (COL3A1), type V collagen *α*_2_ chain (COL5A2), and periosteal protein (POSTN).

### 3.4. Prognostic Values of Hub Genes

To evaluate the prognostic values of 5 hub genes above identified in BC, we mapped them into the Kaplan–Meier database for their correlations with BC survival, with the log-rank test and a 95% hazard ratio (HR) calculated. Among these 5 hub genes, we found the expressions of COL1A1 [HR= 0.72 (0.58–0.91), *P*=0.005], COL3A1 [HR= 1.28 (1.02–1.6), *P*=0.031], and POSTN (HR= 0.75 (0.6–0.94), *P*=0.031) were significantly correlated with overall survival of BC patients (Figure 4), while the expressions of LUM [HR= 0.82 (0.66–1.03), *P*=0.084] and COL5A2 [HR= 0.95 (0.76–1.19), *P*=0.66] were not.

## 4. Discussion

A wealth of supporting evidence indicates that the incidence rate of BC is increasing year by year, especially among young women, posing a serious threat to women's physical and mental health and global public health issue [13, 14]. In the advanced stage, BC patients often suffered from cancer metastasis, leading to poor prognosis. BM is one of the causes of high mortality in patients with BC [15]. Furthermore, the patients with advanced BC have a high recurrence rate even if they have been cured. Therefore, early screening strategies would lead to more effective treatments for BC patients with BM and lower the risk of developing BM.

With the development of genomics and bioinformatics, BC-related data are available in many databases, which provide valuable information for us to identify new biomarkers of BC patients with BM [16, 17]. In our study, two datasets including GSE125989 and GSE100534 were applied to identify DEGs between primary BC samples and BM samples, and then 19 overlapped DEGs were observed using the Venn diagram, including COL1A1, DPT, GREM1, CILP, POSTN, IGF1, COL3A1, THBS2, COL14A1, LUM, ACTA2, COL6A3, LRRC15, CCL19, MMP11, COL5A2, AOX1, KRT14, and GAP43. Neoplastic cells are considered as a critical element for BC development and progression. Recent studies indicated that alterations in the surrounding stroma and components of the tumor microenvironment, such as suppressive immune cells and soluble factors, regulated BC progression and metastasis [18, 19]. Indeed, some key genes are involved in this process. Tan et al. [20] revealed that proto-oncogene Erbb2 was overexpressed in breast cancer cells and highly associated with pulmonary metastasis. Lee et al. demonstrated that SOX2 and OLIG2 genes were upregulated in BC patients with BM [21]. An in-depth understanding of the functional role of DEGs is of great significance for identifying therapeutic biomarkers related to cancer metastasis. Cancer cells usually exhibit antiapoptosis ability, which is a prerequisite for cancer cell metastasis and diffusion. The extracellular matrix affects cancer cell characteristics and is related to cell metastasis [22]. The ECM structural constituent, ECM organization, and collagen catabolic process might be responsible for the occurrence of BM in BC patients [23]. In the present study, we conducted GO annotation and KEGG pathway analyses on 19 overlapped DEGs between primary BC and BM samples. It was found that these DEGs were mainly enriched in GO terms such as extracellular matrix organization, extracellular structure organization, and tissue regeneration. In addition, we observed that 6 signal pathways, including protein digestion and absorption, focal adhesion, ECM-receptor interaction, relaxin signaling pathway, the PI3K-Akt signaling pathway, and proteoglycans in cancer, were confirmed by KEGG pathway analysis. Activation of various signaling pathways, such as STAT3 signaling pathway and PI3K-Akt signaling pathway, is related to metastasis in both BC cells and the tumor microenvironment [24]. Blazquez et al. manifested that the protein expression of the PI3K signaling pathway in some BM samples of BC is limited to the microenvironment [25]. Activation of PI3K-Akt signaling contributed to bad outcomes in patients with BC and BM [26, 27]. Some key genes were found to be linked with overall survival of BC in some research works. ANLN, BUB1, TTK, and SKA3 affected overall survival of BC patients [28]. Overexpression of genes consisting of COL1A1, COL14A1, COL5A1, COL6A1, and COL6A2 were unfavorable for prognosis of BC patients metastasized to the brain [23]. In our study, the first five hub genes screened through the PPI network, including COL1A1, LUM, COL3A1, COL5A2, and POSTN, were associated with BC survival. There was a close correlation between three hub genes (COL1A1, COL3A1, and POSTN) and overall survival of BC patients. These findings were supported by other studies to an extent. Liu et al. pointed out that COL1A1 silencing inhibited metastasis of BC cells and achieved a better survival [29]. In triple-negative BC, METTL3 suppressed the metastasis of cancer cells via decreasing expression of COL3A1 and the increasing m6A level [30]. POSTN overexpression observed in various cancer types including BC is correlated with metastasis and tumor progression [31].

Some limitations, of course, existed in our study. Firstly, this study was performed only based on the bioinformatics analysis of published datasets in the absence of corresponding experimental verification. Secondly, we can predict the most relevant genes leading to BM in cancer patients by the logistic regression model, further identifying crucial genes for occurrence of BM. Finally, the sample size from two datasets was relatively small, which might cause bias of the results. In general, this study identified 5 hub genes potentially related to BC patients with BM through a series of bioinformatics analysis, and COL1A1, COL3A1, and POSTN genes were significantly associated with overall survival of BC patients. These data would provide insights into the development of novel biomarkers for BC patients and the diagnosis along with prognosis of BC patients suffering from BM.

## Figures and Tables

**Figure 1:** Identification of DEGs in BC associated with BM. (a) The volcano plot and heatmap showing DEGs between primary BC and BM samples after analyzing the GSE125989 dataset. (b) The volcano plot and heatmap showing DEGs between primary BC and BM samples after analyzing the GSE100534.

**Figure 2:** Functional enrichment analysis of DEGs. (a) Venn diagram analysis showed 19 overlapped DEGs containing an overlapped upregulated DEG and 18 overlapped downregulated ones. (b) GO analysis of DEGs between primary BC and BM samples. (c) KEGG pathway analysis of DEGs between primary BC and BM samples.

**Figure 3:** DEGs between primary BC and BM samples into the STRING online tool to construct a PPI network.

**Figure 4:** COL1A1, COL3A1, and POSTN were mapped them into the kaplan-meier database and found to be correlated with BC survival.

## Data Availability

The data used to support the findings of this study are included within the article.
